# Analysis of the Mechanism of Ureproofing Technology and Postlaparoscopy on Patients with Urology and Infection

**DOI:** 10.1155/2022/4373416

**Published:** 2022-04-21

**Authors:** Si Chen, Yuanfeng Zhang, Peilin Shen, Zhuangcheng Huang, Mingen Lin, Jiansheng Huang

**Affiliations:** ^1^Department of Urology, The First Affiliated Hospital of Shantou University Medical College, Shantou, Guangdong 515041, China; ^2^Department of Urology, Shantou Central Hospital, Shantou, Guangdong, China

## Abstract

**Objective:**

To analyze the effect of ureteroscopy and retrolaparoscopy on urinary calculi and infection.

**Method:**

A total of 64 patients with urinary calculi and infection who received treatment in our hospital from June 2018 to January 2018 were selected. According to the different treatment methods, they were divided into two groups: a control group and a study group. The study group was treated with laparoscopic ureteroscopy, and the control group was treated with ureteroscopy. The surgical results, complications, renal function, stress response, and inflammatory reaction were compared between the two groups.

**Results:**

Compared with the control group, the study group stone clearance rate was higher, the surgical time was shorter (*P* < 0.05); the incidence of complications in the study group (23.3%) was lower than that in the control group (5.9%) (*P* < 0.05); there was no significant difference in kidney function indicators before treatment (*P* > 0.05); after treatment, the SCR, BUN, NGAL, and Cys-C indicators of the two groups were significantly increased. Compared with the control group, the study group change was more obvious, and the difference was statistically significant (*P* < 0.05); after treatment, the two sets of stress response indicators were significantly increased, but relative to the control group, the study group stress response indicator was lower (*P* < 0.05); before treatment, there was no significant difference in inflammatory factors (*P* > 0.05); after treatment, the two sets of inflammatory factor levels were significantly increased, but relative to the control group, the study group was lower (*P* < 0.05).

**Conclusion:**

In the clinical treatment of urinary stones, ureteroscopy technology and the laparoscopic technique have played an important role. But the laparoscopic technique is shorter, the stone clearance is higher, and the patient's renal function can be improved, and the patient is postoperative. The stress reaction should be small. Therefore, in the clinical treatment of urinary stones and infection, laparoscopic technical treatment is worth promoting.

## 1. Introduction

The ureter, urethra, and bladder are prone to highly pathogenic disease, and the clinical treatment of ureteral calculi is focused on [1]. Data show that about 70% of ureteral stones can be passed naturally. If the past medical history is large, it is difficult to discharge naturally [2]. At present, urological equipment is becoming more and more advanced, surgical technology is improving, and ureteroscopy and laparoscopy have been widely used [3].

Due to the ureteral mirror crimping stone, the stone residue is prone to stones, but the laparoscopic urinary tube is cut into the ureteral tour at the stone, and the ureteral expansion is blocked above the stone, and there will be little stone residual phenomenon [4, 5]. However, the current research on the safety and mechanism of the abovementioned two treatment methods is limited. The study selection included 64 cases of urinary stones admitted to our hospital from June 2018 to January 2021, and the abovementioned two methods were selected. The report of the analysis of the treatment effects of urinary stones in infected patients is further discussed in this study.

## 2. Data and Methods

### 2.1. General Information

A total of 64 patients with urinary tract stones complicated by infection who were treated in our hospital from June 2018 to January 2018 were selected and divided into the control group and the study group according to different treatment methods. The study group (*n* = 34) had 18 males and 16 females with an average age of 48.5 ± 5.5; the control group (*n* = 30) had 16 males and 14 with an average age of 48.3 ± 5.6. This study was approved by the patients' consent and the hospital ethics committee, and the data were comparable (*P* > 0.05).

 
*Inclusion Criteria*: (1) age of 20–72; (2) imaging and clinical diagnosis of CT and ultrasound, diagnosed as urinary stones and infected; (3) acceptable forecast follow-up; and (4) high quality, which can be combined with the researcher
 
*Exclusion Criteria*: (1) congenital ureteral narrow malformation; (2) urinary tuberculosis and ureterodialysis; (3) combined with hemorrhagic diseases; (4) hepato cutter is abnormal; (5) kidney damaged features due to consolidation of severe renal water; and (6) surgical contraindications

### 2.2. Method

1. Laparoscopic ureterotomy: the patient is placed in a supine position, tracheal intubation is anesthetized, and the dilated ureter bursts at the extraction site of the lower part of the kidney, which can be freely descended. The ureter is clamped by the separation clip, the electric hook is removed longitudinally, the ureter is cut off, and the stone is taken out. The 5f double-J tube was inserted through the proximal and distal ends of the ureteral incision, and absorbable sutures were selected to suture the ureteral incision, leaving the abdominal drainage tube.
2. Ureteroscopic lithotripsy: the patient was placed in a supine position, and the back was anesthetized with hard lumbar anesthesia, and an 8/9.8F ureteroscope was placed in the urethra. Under the guidance of a zebra wire, it is placed into the patient's ureter to control the appropriate perfusion pressure. After the stone was detected, the holmium laser 400 *μ*m fiber had reached the catheter, and the edge of the stone was gradually crushed. Finally, the retrograde 5F double J tube.

### 2.3. Observation Indicator

 
*Surgical Results*: it includes the operation time, hospitalization time, postoperative analgesic pump, calculi clearance rate, and polyps discovery rate
 
*Complications*: statistical ureteral vacation, fever, incision infection patients, and calculation incidence
 
*Renal Function* [6]: 3 ml of venous blood is taken, centrifuged at 3000 rpm for 10 minutes, and an automatic biochemical analysis of serum, serum creatinine (SCR), blood urea nitrogen (BUN), and apolipoprotein (NGAL) indicators instrument (Ponzi Medical, model: PUZS-300X) is used and operated according to the instruction manual
 
*Stress Reaction* [7]: serum tyrosinase (NE), adrenal hormone (ACTH), cortical hormone (COR) index, application of enzyme-linked immunosorbent assay (ELISA), and fat were provided by American Beckman Box, and the operation was carried out according to the instruction manual
 
*Inflammatory Reaction* [8]: application of immunimosis for the detection of C-reactive protein (CRP), automatic biochemical analyzer is applied to detect white blood cells (WBCs), application of the enzyme immunization adsorption method to detect interleukin-10 (IL-10)

### 2.4. Statistical Method

The data were analyzed and processed by SPSS22.0 statistical software. The quantitative data were represented by the mean ± standard deviation, the *T* test was performed, group data were analyzed by variance, the *X*^2^ test was used for qualitative data, two-sided test statistics were used, and *P* < 0.05 was different; graphs were used. Rates were made by GraphPad Prism 8, *P* < 0.05 was significantly different.

## 3. Results

### 3.1. General Data Analysis of Two Groups

In the control group and research group, gender, age, preoperative culture positive, and preoperative indwelling double J tube rate, there is a statistical significance (*P* > 0.05) (Table 1).

### 3.2. Surgical Results of Two Groups Were Analyzed in Two Groups of Hospitalization Time

The time of use of postoperative analgesia did not show a significant difference (*P* > 0.05). In the control group and the study group, the stone clearance was 81.7% and 100%, respectively. In comparison, the stones of the study group were higher, the surgical time was shorter, and there was statistical significance (*P* < 0.05) (Table 2).

### 3.3. Comparison of Complications between the Two Groups

The incidence of complications in the study group was lower than that in the control group (Figure 1).

### 3.4. Two-Group Kidney Function Index Contrast

Before the analysis of kidney function indicators, the two groups of renal function indicators have no significant difference (*P* > 0.05). After treatment, SCR, BUN, NGAL, and Cys-C indicators of two groups were significantly increased. Compared with the control group, the study group change is more obvious, and there is a statistical significance of the difference (*P* < 0.05) (Figure 2).

### 3.5. Comparison of Two Groups of Oxidative Stress Indicators

There was no significant difference in oxidative stress indicators between the two groups (*P* > 0.05), and the stress response indicators in the two groups were significantly increased after treatment, which should be higher in the study group than in the control group (*P* < 0.05) (Figure 3).

### 3.6. Comparison of Inflammatory Response Indexes between the Two Groups

There was no significant difference in inflammatory factors between the two groups before treatment (*P* > 0.05), and after treatment, the inflammatory factors in the two groups were significantly increased, but compared with the control group, the study group was lower (*P* < 0.05) (Figure 4).

## 4. Discussion

The treatment of ureteral calculi is particularly special, and open surgery, ureteroscopy, laparoscopy, and transdermal nephroscopy are often used [9–11]. Minimally invasive surgery is used if the patient has contraindications to traditional surgery [12, 13]. At present, laparoscopy and ureteroscopy have been widely used in the treatment of urology, and ureteroscopic lithotripsy can be operated according to the characteristics of the human body's natural cavity and low wound surface. Combined with laser treatment, it can effectively crush stones. Stenosis can be treated concurrently, but ureteral stones are less effective [14, 15]. The main reasons are that the ureteral walker is long, stones are often used by ureteral budding polyps, and factors such as ureteral transformation will also affect the treatment effect. The high rate of ureteral perforation and tearing enables the clinical treatment of ureteral mirror crimping stones [16, 17]. Therefore, when choosing the treatment method for ureteral calculi, the situation of the distal ureter should be comprehensively analyzed. Ureteroscopy is widely used in the treatment of larger ureteral calculi, and the treatment effect is good and the safety is relatively high [18]. After the end of the study, the patients were treated with ureteroscopy. No obvious complications were found, and the prognosis of the patients was good [19]. During ureteroscopy treatment, stone movement is common, and the following measures can be taken to reduce the incidence of stones on stones. The patient's position is lower than their head [20]. Second, perform low-pressure perfusion during operation, maintaining low-speed flushing. Third, when placing the ureteral stent, the edge should be placed on the edge of the stone and should be pressed to the ureteral side [21]. Fourth, when selecting cases, the specific characteristics of the patients should be considered, and patients with a combined case with a stone diameter greater than or equal to 1.0 cm, a fixed stone, and a longer course of disease should be selected [22].

In urology, laparoscopy has been widely used, which has accelerated the progress of ureteral diameter technology. It has the characteristics of fast postoperative recovery and small damage, which can make up for the defects of traditional open surgery and be used for the treatment of ureteral stones [23]. Laparoscopic urinalysis can complete one-time stones, but laparoscopy is skilled. In this study, laparoscopy was used to treat patients with ureteral calculi, and the effect was satisfactory, with a stone clearance rate of 100% and a shorter operation time [24]. This study analyzed the effects of ureteroscopy and laparoscopy on the prognosis of patients with urinary calculi and infections. The incidence of complications was consistent with the findings of other scholars. The results confirmed that laparoscopic urinary tandem resection had lower complication rates and higher surgical success rates compared with ureteroscopic culprits. Surgery is an invasive treatment, which will stimulate the body to a certain extent. The patient will be accompanied by stress, and the immune function of the patient will be reduced, which will affect the postoperative recovery. Among them, the activation of the hypothalamus-pituitary-adrenal axis is mainly due to the stress response, and the amount of Ne, ACTH, COR, and other hormones increases significantly, which can reflect the stress state of the body [25]. This study analyzed the effects of ureteroscopy and postlaparoscopic techniques on stress response indicators in patients with urinary calculi and infection. The results showed that the stress response indexes of the two groups were significantly increased after treatment, but compared with the control group, the stress response indexes of the study group were lower (*P* < 0.05). The results confirmed that after reducing the stress response, the advantages of laparoscopic technology were more obvious, causing less damage to the patient and speeding up the recovery of the disease.

However, after the laparoscopic urine test, pay attention to the following aspects: (1) accurately locate by X-ray mode before operation, determine the anatomical signs such as calculus, kidney compression, lumbar bust, and peritoneum, and explore the ureter. (2) The cutter is held over the stone with breakaway pliers to prevent mobilization of the stone [26]. (3) Shorten the time of the double J tube. After the double J tube is placed, the ureteral catheter needs to be removed. The development of medical technology after the laparoscopic urine test has the possibility of shortening [27].

## 5. Conclusion

In the clinical treatment of urinary stones, ureteroscopy technology and the laparoscopic technique have played an important role, but the laparoscopic surgery time is shorter, and the stone clearance rate is higher, and the patient's renal function can be improved to a greater degree of kidney function. The patient's stress reaction should be small after surgery. Therefore, in the clinical treatment of urinary stones and infection, laparoscopic technical treatment is worth promoting.

## Figures and Tables

**Figure 1:** Comparison of complications between the two groups.

**Figure 2:** Two-group kidney function index contrast.

**Figure 3:** Comparison of two groups of oxidative stress indicators.

**Figure 4:** Comparison of inflammatory response indexes between the two groups.

**Table 1:** Analysis of the general data of two groups.

Project	Control group (*n* = 30)	Research group (*n* = 34)	*X* ^2^/*t*	*P*
Gender (male/female)	16/14	18/16	0.682	＞0.05
Age	48.3 ± 5.6	48.5 ± 5.5	1.524	＞0.05
Preoperative urine culture positive (example, %)	5 (16.7)	5 (14.7)	0.638	＞0.05
Introduction double J tube (example, %) before surgery	20 (66.7)	23 (67.6)	1.724	＞0.05

**Table 2:** Analysis of the surgical results of the two groups.

Group	Count	Surgery time (min)	Hospital stay (day)	Postoperative analgesia pump usage time (D)	Stone clearance (%)	Polyps discovery rate (%)
Control group	30	49.3 ± 7.8	5.2 ± 1.4	2.2 ± 0.6	49 (81.7)	33 (55.0)
Research group	34	41.4 ± 5.4	5.1 ± 1.3	2.3 ± 0.5	68 (100.0)	37 (54.4)
*X* ^2^	—	17.625	1.082	1.824	5.638	0.724
*P*	—	＜0.05	＞0.05	＞0.05	＜0.05	＞0.05

## Data Availability

The data used to support the findings of this study are available from the corresponding author upon request.
